# Is It Compartment Syndrome? Two Case Reports and Literature Review

**DOI:** 10.7759/cureus.19083

**Published:** 2021-10-27

**Authors:** Hasan Aleisawi, Ghadeer Alsager, Abdulrahman Pasha, Hussain Alyousif, Hani Alsarhan, Saad Surur

**Affiliations:** 1 Orthopaedic Surgery, King Saud Medical City, Riyadh, SAU

**Keywords:** fasciotomy, acute compartment syndrome, trauma, intracompartmental pressure measurement, fracture

## Abstract

Recently, a unique entity of acute compartment syndrome (ACS) has been termed “silent” compartment syndrome. These patients develop ACS in the absence of classic pain and physical findings. We report two cases of posttraumatic silent ACS in two healthy competent adult patients presenting mainly with swollen tense compartments. In the first case, ACS was suspected in a 37-year-old male with left tibia and fibula shaft fractures after reassessment of the patient’s post-backslap application, which revealed painless swollen and tense compartments. In the second case, ACS suspicion was raised in a 27-year-old male with right comminuted tibial plateau fracture and a swollen but soft compartment that became tense over time. In both cases, intraoperative intracompartmental pressure testing during external fixator application confirmed the diagnosis, and both underwent emergent fasciotomy with good postoperative outcomes. The absence of pain does not exclude the diagnosis of ACS. Physicians must have a high index of suspicion when risk factors are present for ACS, and the diagnosis can be confirmed with intracompartmental pressure measurement. These case reports and literature review aim to enlighten the physicians about silent compartment syndrome.

## Introduction

Acute compartment syndrome (ACS) is a clinical entity that can be defined as “an elevation in interstitial pressure in a closed fascial compartment that results in microvascular compromise. As the duration and magnitude of the pressure increase, myoneural function is impaired, and necrosis of the soft tissue eventually develops” [1]. ACS is currently considered a clinical diagnosis. A tense swollen limb, pallor, paresthesia, paralysis, and pulselessness are signs of underlying ischemia, but these signs and symptoms are poor predictors of the occurrence of ACS [2,3]. The presence of concomitant nerve injuries with loss of sensation, altered level of consciousness, the effect of anesthesia, and conditions that render patients incompetent may mask the diagnosis of ACS. However, in neurologically responsive, sensate, and competent patients, the development of pain that is out of proportion to the injury and that is not relieved by analgesia is traditionally considered to be the earliest, most sensitive, and reliable indicator of the development of an underlying compartment syndrome [4,5].

Herein, we report two unique cases of compartment syndrome in competent and sensate patients. We also performed a literature review, and discussed the diagnosis and implications.

## Case presentation

Case 1

A 37-year-old healthy male patient was brought to the emergency department (ED) after a side collision of his motor vehicle with a truck at 15:00. On arrival, the patient was hemodynamically stable and was found to have an isolated left lower limb injury. Upon examination by the on-call orthopedic specialist at 22:00, the patient had a deformed left leg and complained of mild pain with tenderness. The visual analogue scale (VAS) score in the ED was 3/10. Assessment of the soft tissue revealed relatively soft compartments. Realignment of the left leg and application of an above-knee backslab were performed. Vascular examination revealed palpable and audible dorsalis pedis and posterior tibial arteries. Radiographs demonstrated left tibia and fibula shaft fractures (Figure 1A, 1B). The patient was comfortable with routine analgesia; after an initial dose of 5 mg of morphine in the ED 30 min after the presentation, he was then put on regular intravenous acetaminophen (1 g) and ibuprofen (400 mg). Re-evaluation of the patient at 06:00 revealed significantly swollen and tense compartments. Because the compartments raised suspicion for ACS, a stretch test was performed and shown to be negative. Although the patient did not have the classic presentation of pain out of proportion to the injury, which is usually associated with ACS, and was comfortable with routine analgesia overnight, he had significantly tense calf muscles, which raised the suspicion of ACS, and the patient was booked for external fixation and possible emergent decompressive fasciotomy.

**Figure 1:** A: Anteroposterior radiograph demonstrating comminuted tibial shaft fracture and proximal fibula fracture. B: Lateral radiograph demonstrating comminuted tibial shaft fracture and proximal fibula fracture. C: Post-operative anteroposterior radiograph showing the placement of an external fixator to the tibial shaft fracture as well as the presence of rubber band lace-up technique on both sides of the leg.

The patient was placed in the supine position under general anesthesia, and the leg was prepped and draped in a standard fashion. Strikingly, large blisters in the fracture area developed rapidly. Because the patient was sensate and competent with unusual and suspicious presentation of acute compartment syndrome, an intraoperative compartment pressure measurement was performed using the arterial line manometer technique. A side-port needle was inserted within 5 cm of the fracture area. The deep posterior compartment measured 89 mmHg, the anterior compartment measured 49 mmHg, the diastolic pressure was 75 mmHg, and the differential pressure was 26 mmHg, confirming the diagnosis of ACS [6,7]. The patient underwent a dual-incision decompressive fasciotomy to decompress all four compartments of the leg. The muscles escaped from the osteofascial compartments, which further confirmed the diagnosis. The superficial and deep posterior compartments showed patchy areas of dusky muscle tissue, but bleeding and contractility. The wounds were partially approximated using a rubber band lace-up technique. Under image guidance, an external fixator was applied to the tibia to provide provisional stability (Figure 1C). In the following week, the patient was subjected to irrigation and debridement, and the wounds were approximated using the rubber band lace-up technique under general anesthesia twice, and during the second time, all wounds were closed. By the end of the week, the patient underwent definitive fixation using an intramedullary nail of the left tibia and percutaneous screw fixation of the proximal tibial split fracture (Figure 2A, 2B). Postoperative examination revealed good range of motion with intact neurovasculature. The patient was discharged with instructions to perform toe touch weight-bearing exercises. At two weeks, the wounds were inspected, and the stitches were removed. At three months, the patient was re-evaluated. He was pain-free, with healed scars, full range of motion of the knee and ankle joints, and did not have any neurological symptoms.

**Figure 2:** Definitive treatment. A: Post-operative anteroposterior radiograph demonstrating definitive fixation of tibial fracture by an intramedullary nail. B: Post-operative lateral radiograph demonstrating definitive fixation of tibial fracture by an intramedullary nail.

Case 2

A 27-year-old healthy male patient presented to the ED with a history of a 3-meter fall during work in which he landed on his feet. Initial clinical examination of the lower extremities at 13:00 showed intact skin and significant right proximal leg deformity associated with swelling and tenderness with a VAS of 3-4/10. Vascular evaluation of distal pulses revealed that the posterior tibial artery pulse was not palpable. The capillary perfusion was less than 2 seconds. The foot was sensate. Initial assessment also revealed swollen but soft compartments; however, the passive stretch test was negative and did not indicate an ACS. Radiographs showed a severely comminuted tibial plateau fracture (Figure 3A). Realignment of the tibial plateau fracture was performed under procedural sedation and an above-knee backslab was applied, followed by reassessment of distal pulses, which showed Doppler-able but weak pulses of the posterior tibial and dorsalis pedis arteries (Figure 3B). Due to the severity of the injury, its natural association with vascular injuries, and the inability to palpate the posterior tibial artery pulses on initial assessment, computed tomography angiography (CTA) was performed, which revealed attenuation of the popliteal artery with patent superficial femoral and anterior and posterior tibial arteries (Figure 3C). The findings were communicated and thoroughly discussed with the on-call vascular surgeon. He concluded that attenuation was not an injury but a compression caused by the posterior tibial plateau and required only serial distal neurovascular assessment. The patient received a dose of fentanyl (50 mg) upon arrival, followed by morphine (5 mg) two hours later, and was then intravenously administered regular doses of acetaminophen (1 g).

**Figure 3:** A: Anteroposterior radiograph demonstrating comminuted tibial plateau fracture associated with dislocation. B: Lateral radiograph after realignment was performed demonstrating comminuted tibial plateau fracture. C: Axial cut of computed tomography scan at the level of both tibial plateau demonstrating comminuted right tibial plateau fracture, and near-total obliteration of the right popliteal artery (red arrow). Additionally, note the presence of significant soft tissue swelling of right leg compared to left leg.

The patient was scheduled for application of a knee-spanning external fixator; however, this was delayed due to two life-saving procedures occupying the operating rooms. Re-evaluation of the compartments in the holding bay at 20:00 revealed quite tense compartments, especially the anterior compartment, but the passive stretch test was negative. Therefore, the patient was consented for a spanning external fixator application with/without fasciotomy of the compartments, depending on the intraoperative compartment pressure measurements. The patient was placed in the supine position under general anesthesia, and a spanning external fixator of the tibial plateau fracture was applied under image guidance (Figure 4A). Compartment pressure testing using the same method revealed a pressure of 66 mmHg within the posterior deep compartment, 54 mmHg in the posterior superficial compartment, 69 mmHg in the anterior compartment, and 45 mmHg in the lateral compartment [6,7]. Therefore, the decision was made to proceed with a decompressive fasciotomy using dual incisions to decompress all four compartments of the leg. Not surprisingly, the anterior compartment muscles significantly escaped when decompressed and were partially dusky with reduced ability to bleed when tested. Irrigation and debridement were performed. The fasciotomy wounds were approximated by the rubber band lace-up technique to keep the skin partially approximated but tension-free. Postoperative examination revealed a perfused limb with capillary refill of less than 2 seconds, and an intact neurological examination; however, distal pulses were not palpable and could not be detected by a hand-held Doppler device. Thus, an urgent CTA was arranged to reveal the patent arteries.

**Figure 4:** Definitive treatment. A: Post-operative anteroposterior radiograph showing the placement of a spanning external fixator to the right knee as well as the presence of rubber band lace-up technique on both sides of the leg. B. Intra-operative anteroposterior flouroscopic view showing definitive fixation of the right tibial plateau fracture. C. Clinical image showing healed scars and good soft tissue status.

Two days later, the patient underwent irrigation, debridement, and wound closure under spinal anesthesia. Finally, the patient underwent open reduction internal fixation with bone graft and plate and screw fixation of the right tibial plateau fracture in the following week (Figure 4B). The patient was discharged with a right below-knee backslab for two weeks, after which it was removed and placed on a hinged brace. At two weeks, the wounds were inspected, and the stitches were removed. At four months, the patient was re-evaluated (Figure 4C). He was pain-free, with healed scars, and a comparable range of motion of the injured knee and ankle joint to the normal contralateral side, without any neurological symptoms. He had mild limitations during moderate-intensity activities.

## Discussion

Pain that is out of proportion to the known injury and increasing analgesic requirements are considered the hallmarks of ACS. The traditional teaching that pain is the cornerstone of the ACS diagnosis might not be accurate and might result in missed compartment syndromes because pain as a symptom is subjective and difficult to measure, and the literature indicates that there are differences among different age groups, sex, and ethnicities [8]. Additionally, Ulmer et al. showed that the classical clinical signs had a sensitivity of 13%-19% and a positive predictive value of only 11%-15%, which are more useful in excluding ACS than to diagnose it as the probability of ACS with one clinical finding was approximately 25%, and the probability was 93% with three clinical findings. Therefore, the absence of pain does not rule out the possibility of compartment syndrome [9].

Recently, a specific entity of ACS has been termed “silent” and is recognized by the development of ACS in the absence of the classic pain that is out of proportion to the known injury in a neurologically responsive, competent, and sensate individual [5]. Silent compartment syndrome is clinically suspected and confirmed by diagnostic methods. It is important to note that silent compartment syndrome is different from occult compartment syndrome, which occurs in an individual who is non-competent, insensate, or distracted.

There are 10 cases of silent compartment syndrome reported in the literature, including the present two cases, with the majority occurring secondary to traumatic tibial fracture. The most common presenting signs in these patients are either swollen tense compartments or reduced sensation. Table 1 summarizes the findings of all cases in the literature.

**Table 1:** Silent compartment syndrome case reports. MVC: motor vehicle collisions; Fx: fracture; IMN: intramedullary nailing; ROM: range of motion; EHL: extensor hallucis longus; EDL: extensor digitorum longus; M3: grade 3 of muscle power according to Medical Research Council classification of motor nerve dysfunction.

Reference	Age (yr)	Diagnosis	Mechanism of injury	Onset of compartment	Presentation	Analgesic requirements	Compartmental pressure measurement (mmHg)	Outcome
Case 1	37	Tibial shaft fx	MVC	Post-trauma	Swollen tense compartments	Morphine (5mg), acetaminophen (1g), & ibuprofen (400mg)	Anterior 49 & deep posterior 89	Good ROM & pain free
Case 2	27	Tibial plateau fx	Fall from 3 m height	Post-trauma	Swollen tense compartments	Fentanyl (50mcg), morphine (5mg), & acetaminophen (1g)	Anterior 69, lateral 45, superficial posterior 54, & deep posterior 66	Good ROM & pain free
Badhe et al. [5]	43	Tibial plateau fx	Fall from 5 m height	Post-trauma	Swollen tense compartments	Routine Analgesia	Anterior 35 & lateral 85	Good ROM & returned to his occupation at 12 weeks post-injury
Badhe et al. [5]	48	Proximal tibia fx	Heavy object fall	Post-trauma	Swollen tense compartments	Subcutaneous morphine (10mg), & regular oral analgesia	Anterolateral 50 & posterior 45	Partial foot drop
Badhe et al. [5]	23	Tibial shaft fx	Sports injury	Postoperatively following IMN	Hypoesthesia in first web space	Routine analgesia	Lateral 70	EHL weakness
Badhe et al. [5]	18	Femoral shaft fx	MVC	8 hours postoperatively (IMN in hemilithotomy) in the contralateral ‘well-leg’ calf muscle	Swollen tense compartment, dull ache in the calf, & decreased urine output with myogloinuria	Morphine (28mg)	Superficial posterior 110 & deep posterior 100	Amputation
Hitz et al. [10]	21	Open tibial shaft fx	MVC	5 days postoperatively (IMN)	Hypoesthesia & foot drop.	Paracetamol & Novaminsulfon	Anterior 80	EHL (M3) and EDL (M3). Pain-free & returned to occupation after 1 year
Wright et al. [11]	39	Fibula head fx	Pedestrian crush injury	Post-trauma	Hypoesthesia & foot drop	Paracetamol (1g) / Codeine phosphate (60mg)	Not measured	Return of sensation and foot dorsiflexion and hallux extension MRC power grade 4/5
Godavitarne et al. [12]	63	Mitral valve regurgitation	Peripheral cannulation of the right femoral vein and artery	Postoperatively	Hypoesthesia	Patient controlled analgesia	Anterior 40, lateral 48, superficial posterior 41, & deep posterior 81	Good
Blanchard et al. [14]	75	Compartment syndrome	Fall	Post-fall	Swollen tense compartments, hypoesthesia, & decreased power in both lower limbs	None	All compartments pressure ranged between (25 and 65 mmHg).	Death

Badhe et al. questioned the reliability of severe pain as an indicator of an underlying compartment syndrome, as they reported silent compartment syndrome in four competent male adult patients, two of which were post-traumatic and two occurred postoperatively. Each patient had a different presentation including mild pain, tense compartments, or hypoesthesia. The patients were treated with emergency fasciotomy with variable outcomes [5]. 

Of the four cases reported by Badhe et al., two cases shared similarities with the present two cases of swollen tense compartments in posttraumatic competent male adult patients with high intracompartmental pressure (ICP) measurements. These occurred in male patients aged 43 and 48 years old following tibial fractures who were comfortable on routine analgesia, and only the presence of swelling and tense compartment raised the suspicion of ACS. After emergent fasciotomy, the first patient had a good follow-up outcome, while the second patient developed a partial foot drop. A third patient developed silent ACS after intramedullary nailing of the tibia. The patient presented with weakness of the extensor hallucis longus and blunting of sensation on the first webspace. The symptoms persisted despite decompressive fasciotomy. The last patient was involved in MVC and sustained high-energy right femoral shaft fracture that was fixed using an intramedullary nail. The patient developed silent compartment syndrome in the contralateral ‘well-leg’ due to hemi-lithotomy position. However, silent compartment syndrome was not suspected until he complained of mild dull ache in the well-leg eight hours post surgery. Later, he underwent amputation [5].

Hitz et al. reported a case of silent ACS five days after post-intramedullary nailing of a tibial fracture. The presentation was a foot drop and reduced sensation in the first webspace, and the patient underwent emergency fasciotomy of all four compartments of the lower leg. Follow-up after a year showed a good outcome, with the patient being pain-free and returning to his occupation after a year [10]. A similar case was presented by Wright et al. in a 39-year-old male who developed foot drop and hypoesthesia in the first webspace following a traumatic fracture of the fibular head. The patient’s neurologic symptoms progressed rapidly without remarkable pain or swelling. He underwent decompressive fasciotomy and, interestingly, his symptoms improved significantly [11].

Godavitarne et al. reported the case of a 63-year-old male with severe mitral valve regurgitation who underwent elective minimally invasive mitral valve repair with peripheral cannulation of the right femoral vein and artery. Twelve hours postoperatively after extubation, the patient reported mild pain in the right lower leg only. On next day, the patient continued to complain of mild right lower leg pain associated with a subjective decrease in sensation. Although, he was prescribed a patient-controlled analgesia (PCA), only one bolus was given. Compartmental pressures were increased significantly. The patient underwent a decompressive fasciotomy of the leg [12]. It is important to note that PCA has been shown delay the diagnosis of acute compartment syndrome, which might lead to unfavorable consequences [13].

Blanchard et al., report an unusual case of a 75-year-old female with atraumatic silent compartment syndrome. She presented to the ED after being unable to rise from a kneeling position for 4 hours. Physical examination revealed swollen legs bilaterally with decreased power and sensation. No significant pain was reported. An ICP measurement was done and a value between 25-65 mmHg was found, leading to a diagnosis of ACS. The patient underwent emergency fasciotomies, her hospital course was complicated with acute renal failure secondary to severe rhabdomyolysis and septic shock, and she passed away two days after admission [14]. 

Because of our experience and awareness of the presence of such a unique and rare entity of acute compartment syndrome, this led to our early recognition and prompt intervention in a timely manner, and disability was prevented in our patients. We report good postoperative outcomes in both patients in terms of pain and range of motion.

ICP is an objective tool that can help confirm diagnosis. The normal resting limb ICP is 10 mmHg [15]. The critical threshold at which decompressive fasciotomy is required is still a topic of debate, ranging from 30-50 mmHg [16,17]. It has been established that individuals have different ICP values due to variations in systemic vascular resistance and perfusion pressure. Whitesides et al. suggested the use of differential pressure or delta pressure (ΔP) to objectively diagnose ACS [6]. ΔP measures the tissue perfusion pressure by calculating the difference between the diastolic blood pressure and the measured compartment pressure. A ΔP of ≤30 mmHg indicates a decrease in tissue perfusion pressure and is diagnostic of ACS. However, by relying on one-time ICP measurements, Whitney et al. found that the method resulted in a 35% false-positive rate for the diagnosis of compartment syndrome in patients with tibial shaft fractures, which resulted in a high rate of unnecessary fasciotomies. More recently, McQueen et al. found the sensitivity and specificity of continuous ICP monitoring to be high, with estimated positive and negative predictive values of 93% and 99%, respectively [18]. ACP is diagnosed when the differential pressure remains <30 mmHg for more than two hours and the pressure trend shows no sign of imminent improvement to a differential pressure above that level.

We propose to extend the silent compartment syndrome definition to include the absence of not only pain, but also pain exacerbated by passive stretch of the involved compartment. With all of that in mind, the questions that should be answered are whether the pain and physical examination findings of patients with suspected ACS are reliable and whether we are overtreating patients with the so-called “silent” compartment syndrome. Undoubtedly, future studies should thoroughly investigate silent compartment syndrome and perhaps using continuous ICP measurement on those patients might reveal new insights.

## Conclusions

Although ACS is largely considered a clinical diagnosis, the absence of pain does not exclude the diagnosis of ACS. Recently, two entities of acute compartment syndromes have been described. The first is 'occult' compartment syndrome which occurs in an individual who is non-competent, insensate, or distracted. The second is 'silent' compartment syndrome which is an ACS that develops in the absence of the classic pain that is out of proportion to the known injury and/or pain exacerbated by passive stretch in a neurologically responsive, competent, and sensate individual. Review of the literature concerning silent compartment syndrome case reports showed that most patients had minimal to mild pain, and tense swollen limb and/or hypoesthesia. Silent compartment syndrome should be suspected in competent adults with risk factors for ACS, even in the absence of pain. Early recognition is important as it prevents the occurrence of avoidable complications. Physicians must have a high index of suspicion, and the diagnosis can be confirmed with intracompartmental pressure measurement.
